The article "Neurotrophins and Neurotrophin Receptors in Proliferative Diabetic Retinopathy" was published in 2013. Journal: PLoS One.

# Neurotrophins and Neurotrophin Receptors in Proliferative Diabetic Retinopathy

**DOI:** 10.1371/journal.pone.0065472

**Published:** 2013-06-07

**Authors:** Ahmed M. Abu El-Asrar, Ghulam Mohammad, Gert De Hertogh, Mohd Imtiaz Nawaz, Kathleen Van Den Eynde, Mohammad Mairaj Siddiquei, Sofie Struyf, Ghislain Opdenakker, Karel Geboes

**Affiliations:** 1 Department of Ophthalmology, College of Medicine, King Saud University, Riyadh, Saudi Arabia; 2 Laboratory of Histochemistry and Cytochemistry, University of Leuven, KU Leuven, Leuven, Belgium; 3 Rega Institute for Medical Research, Laboratory of Molecular Immunology and Laboratory of Immunobiology, University of Leuven, KU Leuven, Leuven, Belgium; University of Florida, United States of America

## Abstract

Neurotrophins (NTs) are emerging as important mediators of angiogenesis and fibrosis. We investigated the expression of the NTs nerve growth factor (NGF), brain-derived neurotrophic factor (BDNF), neurotrophin-3 (NT-3), and neurotrophin-4 (NT-4) and their receptors TrkA, TrkB, and TrkC in proliferative diabetic retinopathy (PDR). As a comparison, we examined the expression of NTs and their receptors in the retinas of diabetic rats. Vitreous samples from 16 PDR and 15 nondiabetic patients were studied by Western blot analysis and enzyme-linked immunosorbent assay (ELISA). Epiretinal membranes from 17 patients with PDR were studied by immunohistochemistry. Rats were made diabetic with a single high dose of streptozotocin and retinas of rats were examined by Western blot analysis. Western blot analysis revealed a significant increase in the expression of NT-3 and NT-4 and the shedding of receptors TrkA and TrkB in vitreous samples from PDR patients compared to nondiabetic controls, whereas NGF and BDNF and the receptor TrkC were not detected with the use of Western blot analysis and ELISA. In epiretinal membranes, vascular endothelial cells and myofibroblasts expressed NT-3 and the receptors TrkA, TrkB and TrkC *in situ*, whereas NT-4 was not detected. The expression levels of NT-3 and NT-4 and the receptors TrkA and TrkB, both in intact and solubilized forms, were upregulated in the retinas of diabetic rats, whereas the receptor TrkC was not detected. Co-immunoprecipitation studies revealed binding between NT-3 and the receptors TrkA and TrkB in the retinas of diabetic rats. Our findings in diabetic eyes from humans and rats suggest that the increased expression levels within the NT-3 and NT-4/Trk axis are associated with the progression of PDR.

## Introduction

Ischemia-induced retinal angiogenesis in association with the outgrowth of fibrovascular epiretinal membranes at the vitreoretinal interface is the pathological hallmark in proliferative diabetic retinopathy (PDR) and often leads to catastrophic loss of vision due to vitreous hemorrhage and/or traction retinal detachment. Vascular endothelial growth factor (VEGF), an endothelial cell mitogen that also enhances vascular permeability, is thought to be the major angiogenic factor in PDR [1]. The key cellular mediator of fibrosis is the myofibroblast, a cell type differentiated form quiescent fibroblasts. Myofibroblasts are contractile cells, characterized by the expression of α-smooth muscle actin (α-SMA), and their presence is a marker of progressive disease. They have the capacity to produce several extracellular matrix components including collagens, and to induce fibrosis [2]. Previous studies have shown that α-SMA-expressing myofibroblasts are the principal cellular components of PDR epiretinal membranes [3].

Neurotrophins (NTs) are a family of structurally and functionally related growth factors that support the growth and differentiation of developing neurons and that maintain neuron survival in the differentiated tissue. NTs include nerve growth factor (NGF), brain-derived neurotrophic factor (BDNF), neurotrophin-3 (NT-3), and neurotrophin-4 (NT-4). NTs mediate their actions by binding to 3 tropomyosin receptor kinases (Trks). NGF binds TrkA, BDNF and NT-4 bind TrkB, and NT-3 binds TrkA, TrkB, and TrkC. In addition, all NTs can bind p75 neurotrophin receptor (p75NTR) with low affinity, enhancing the activation of Trk receptors [4]. NTs and their corresponding receptors are not only expressed within the nervous system, but are also expressed and functionally active in several non-neuronal tissues [5]–[11]. Although well-known as regulators of neuronal survival, differentiation, and regeneration, NTs have only recently been proposed to be important mediators in the angiogenic process, in addition to the well established role of angiogenic growth factors, such as VEGF. NTs may act directly on local Trk-expressing endothelial cells and on recruited specific subsets of Trk-expressing bone marrow-derived hematopoietic cells or indirectly via induction of pro-angiogenic factors, such as VEGF [5], [12]–[17]. In addition, in several studies it has been shown that NTs modulate several fibroblast functions [6], [8], [18], are able to promote tissue remodeling, and play a role in inflammatory responses, wound healing, and fibrosis [8], [9], [10].

In view of the emerging evidence for the angiogenic and fibrogenic activities of NTs, we investigated the expression of NTs and their receptors in the vitreous fluid and epiretinal membranes from patients with PDR. In addition, we investigated the expression of NTs and their receptors in the retinas of diabetic rats.

## Materials and Methods

### Vitreous Samples and Epiretinal Membranes Specimens

Undiluted vitreous fluid samples (0.3–0.6 ml) were obtained from 16 patients with PDR during pars plana vitrectomy. The indications for vitrectomy were tractional retinal detachment, and/or nonclearing vitreous hemorrhage. The control group consisted of 15 patients who had undergone vitrectomy for the treatment of rhegmatogenous retinal detachment with no proliferative vitreoretinopathy. Controls were free from systemic disease. Vitreous samples were collected undiluted by manual suction into a syringe through the aspiration line of vitrectomy, before opening the infusion line. The samples were centrifuged (500 rpm for 10 min, 4°C) and the supernatants were aliquoted and frozen at −80°C until assay.

Epiretinal fibrovascular membranes were obtained from 17 patients with PDR during pars plana vitrectomy for the repair of tractional retinal detachment. The severity of retinal neovascular activity was graded clinically at the time of vitrectomy using previously published criteria [19]. Neovascularization was considered active if perfused new vessels on the retina or optic disc were present within tractional epiretinal membranes. Neovascularization was considered inactive (involuted) if only nonvascularized white fibrotic epiretinal membranes were present. Active PDR was present in 8 patients and inactive PDR was present in 9 patients. Membranes were fixed in 10% formalin solution and embedded in paraffin.

The study was conducted according to the tenets of the Declaration of Helsinki. All the patients were candidates for vitrectomy as a surgical procedure. All patients signed a preoperative informed written consent and approved the use of the excised epiretinal membranes and vitreous fluid for further analysis and clinical research. The study design and the protocol was approved by the Research Centre and Institutional Review Board of the College of Medicine, King Saud University.

### Rat Streptozotocin-induced Diabetes Model

All procedures with animals were performed in accordance with the ARVO statement for the use of animals in ophthalmic and vision research and were approved by the institutional animal care and use committee of the College of Pharmacy, King Saud University. Adult male Sprague-Dawley rats, 8–9 weeks of age weighting in the range of 250–300 g were overnight fasted and streptozotocin (STZ) (65 mg/kg in 50 mM sodium citrate buffer, pH 4.5, Sigma, St.Louis, MO) was injected intraperitoneally. Equal volumes of citrate buffer were injected in control non-diabetic animals. Measurement of blood glucose concentrations and body weight were started 3 days after injection of STZ. Diabetes was confirmed by assaying the glucose concentration in blood taken from the tail vein. Rats with glucose levels >250 mg/dl were categorized as diabetic. After 12 weeks of diabetes, animals were anesthetized by intraperitoneal injection of an overdose of chloral hydrate and sacrificed by decapitation. Retinas were dissected, flash frozen and stored at −70°C until use. Similarly, retinas were obtained from age-matched nondiabetic control rats.

### Western Blot Analysis

To determine the NGF, BDNF, NT-3,NT-4,TrkA, TrkB and TrkC protein levels in the retinas of 8 non-diabetic and 8 diabetic rats, retinal tissues were homogenized in a Western lysis buffer (30 mM Tris-HCL, pH 7.5, 5 mM EDTA, 1% Triton X-100, 250 mM sucrose, 1 mM Sodium Vanadate and protease inhibitor cocktail). The protease inhibitor used was “Complete without EDTA” (Roche, Mannheim, Germany). The lysate was centrifuged at 14,000×g for 15 min (4°C) and the pellets were removed. The protein concentrations in the supernatants were estimated using the Bio-Rad protein assay kit (Bio-Rad Laboratories Inc., Hercules, CA). Protein samples were boiled in Laemmli’s sample buffer for 10 min and equal amounts of protein (40–50 µg) were separated on 8–15% SDS-polyacrylamide gels (SDS-PAGE) and transferred onto nitrocellulose membranes. To determine the expression levels of NGF, BDNF, NT-3, NT-4,TrkA, TrkB and TrkC in the vitreous samples, equivalent original volumes of vitreous samples (from diabetic or control humans or rats) were boiled in Laemmli’s sample buffer (1∶1, v/v) for 10 min under reducing conditions for BDNF, NT-4, TrkB and TrkC and under non-reducing conditions for NT-3 and TrkA. Equal volumes of lysis solution (15 µL) were loaded and separated on 8–15% SDS-PAGE gels and transferred onto nitrocellulose membranes. The breakdown of the blood-retina barrier leads to raised protein levels in the vitreous fluid of diabetic patients. Therefore, we also determined the levels of NT-3 and TrkA in equivalent amounts of protein (20 µg) from vitreous and paired serum samples obtained from 12 patients.

After protein transfer, the membrane was blocked (1.5 h, room temperature) with 5% non-fat milk and then incubated overnight at 4°C with goat polyclonal anti-NGF (1∶300, Cat No: AF-256NA, R&D Systems, Minneapolis, MN), mouse monoclonal anti-BDNF (1∶300, Cat No: MAB-248, R&D Systems), goat polyclonal anti-NT-3 (1∶300, Cat No: AF-267NA, R&D Systems), goat polyclonal anti-NT-4 (1 µg/ml, Cat No: AF-268, R&D Systems), mouse monoclonal anti-TrkB (1 µg/ml, Cat No: MAB-397, R&D Systems), mouse monoclonal anti-TrkA (1 µg/ml, Cat No: MAB-367, R&D Systems) and rabbit polyclonal anti-TrkC (1 µg/ml, Cat No: ab-75174, Abcam, UK). After incubation with the specified primary antibodies, the membranes were washed and incubated at room temperature for 1.5 h with their respective secondary horseradish peroxidase-conjugated antibody. Membranes were again washed four times and the immunoreactivity of bands was visualized on a Chemi-DocXRS^+^ system (Bio-Rad Laboratories Inc.) with the use of enhanced chemiluminescence and Western blotting luminol reagents (1∶1 v/v, Cat No: SC-2048, Santa Cruz Biotechnology, Inc., Santa Cruz, CA). By densitometric analysis using Image-Lab 2.0.1 software (open source, Bio-Rad Laboratories Inc.), we quantified the protein bands. For internal control, membranes were stripped and incubated with a mouse monoclonal anti-β-actin antibody (1∶2000, Santa Cruz Biotechnology, Inc.) and all remaining steps were followed as detailed above.

### Enzyme-linked Immunosorbent Assay for NGF and BDNF

Enzyme-linked immunosorbent assay (ELISA) kits for human BDNF (Quantikine Brain Derived Neurotrophic Factor, Cat No.: DBD00) and human NGF (Nerve Growth Factor, Cat No: DY256) were purchased from R&D Systems. The detection limit for BDNF was 20 picograms per mL (pg/mL). The ELISA plate readings were done with the use of a FLUOstar Omega-Microplate reader from BMG Labtech (Offenburg, Germany). For each ELISA kit, the undiluted standard served as the highest concentration and calibrator diluents served as the blank. Undiluted vitreous samples were directly used in each ELISA experiment. For the measurements of BDNF and NGF, 50 µL and 100 µL of undiluted vitreous samples were added into each of the respective ELISA plates for the analysis. Following sample incubation, secondary antibodies against BDNF and NGF, conjugated to horseradish peroxidase were added to each well of the ELISA plates. After incubation, substrate mix solution was added for colour development. The reaction was stopped by the addition of 2N sulfuric acid and the optical density was determined at 450 nm in a microplate reader. Each assay was performed in duplicate. With the use of a 4-parameter fit logistic curve equation, the actual concentration for each sample was calculated.

### Immunohistochemical Staining

Endogenous peroxidase was abolished with 2% hydrogen peroxide in methanol for 20 min, and nonspecific background staining was blocked by incubating the sections for 5 min in normal swine serum. Antigen retrieval was performed by boiling the sections in 10 mM citrate buffer [pH 6] for 30 min. Subsequently, the sections were incubated with the monoclonal and polyclonal antibodies listed in Table 1. Optimal working concentrations and incubation times for the antibodies were determined earlier in pilot experiments. The sections were then incubated for 30 minutes with immunoglobulin conjugated to peroxidase-labeled dextran polymer [EnVision (Flex), Dako, Carpinteria, CA, USA]. The reaction product was visualized by incubation for 10 minutes in 0.05 M acetate buffer at pH 4.9, containing 0.05% 3-amino-9-ethylcarbazole (Sigma-Aldrich, Bornem, Belgium) and 0.01% hydrogen peroxide, resulting in bright-red immunoreactive sites. The slides were then faintly counterstained with Harris hematoxylin. Omission or substitution of the primary antibody with an irrelevant antibody from the same species and staining with chromogen alone were used as negative controls. Sections from patients with glioblastoma were used as positive controls for the immunohistochemical staining methods. The sections from the control patients were obtained from patients treated at the University Hospital, University of Leuven, Belgium, in full compliance with tenets of the Declaration of Helsinki. We used archived material and patients gave written consent at admission for the use of the leftover material in studies. The Ethics Committee of the University Hospital, University of Leuven approved this consent procedure.

**Table 1:** Monoclonal and polyclonal antibodies used for immunohistochemical staining.

Primary Antibody	Dilution	Incubation Time	Source*
• Anti-CD34 (Clone My10) (mc)	1/50	60 minutes	BD Biosciences
• Anti- α-Smooth muscle actin (Clone 1A4) (mc)	1/200	60 minutes	Dako
• Anti- Neurotrophin 3 (Catalogue No. ab65804) (pc)	1/100	60 minutes	Abcam
• Anti-Neurotrophin 4 (Catalogue No. ab87394) (mc)	1/50	60 minutes	Abcam
• Anti-TrkA (763): SC-118 (pc)	1/50	60 minutes	Santa Cruz Biotechnology, Inc.
• Anti-TrkB (H-181): SC-8316 (pc)	1/50	60 minutes	Santa Cruz Biotechnology, Inc.
• Anti-TrkC (798): SC-117 (pc)	1/100	60 minutes	Santa Cruz Biotechnology, Inc.

* Location of manufacturers: BD Bioscience, San Jose, CA, USA, Dako, Glostrup, Denmark, Abcam, Cambridge, UK, Santa Cruz Biotechnology, Inc., Santa Cruz, CA, USA.

mc = monoclonal, pc = polyclonal.

### Quantitation

Immunoreactive blood vessels and cells were counted in five representative fields, using an eyepiece calibrated grid in combination with the 40×objective. These representative fields were selected based on the presence of immunoreactive blood vessels and cells. With this magnification and calibration, immunoreactive blood vessels and cells present in an area of 0.33×0.22 mm^2^ were counted.

### Co-immunoprecipitation

Retina tissue was homogenized in 30 mM Tris-HCl lysis buffer, pH 7.5 containing 10 mM EGTA, 5 mM EDTA, 1% Triton X-100, 250 mM sucrose, 1 mM NaF, 1 mM phenylmethylsulfonyl fluoride and 1 mM Na_3_VO_4_. Protein (120µg) was incubated overnight at 4°C with 2 µg of anti-NT-3 antibody. Agarose beads A/G (Santa Cruz Biotechnology, Inc.) were washed with lysis buffer, and were mixed with the lysates for 1 h at 4°C to capture NT-3 immune complexes. Samples were boiled in Laemmli buffer and subjected to electrophoresis on SDS-PAGE. Western blot analysis was performed using antibodies against TrkA and TrkB.

### Extracellular Signal-regulated Kinase (ERK) Signaling Assay

Phosphorylation of ERK 1 and ERK 2 was analyzed in human retinal microvascular endothelial cells (HRMEC, Cell Systems, Kirkland, WA) as previously described [20]. HRMEC were cultured in endothelial basal medium-2 (EBM-2) enriched with endothelial growth medium-2 MV Bulletkit (Lonza, Verviers, Belgium). Cells were seeded in 6-well plates at 15000 cells/cm^2^. At a confluency level of 80% or more, cells were starved from growth factors by replacing their growth medium with EBM-2 without any supplements. After being deprived of growth factors overnight, the starvation medium was replaced with EBM-2, supplemented with 0.5% Bovine Serum Albumin (BSA) (Sigma-Aldrich) at least 15 min prior to induction. Ten-fold dilutions of the inducers [NT-3, NT-4 or VEGF, all from R&D Systems] were prepared in the EBM-2/BSA medium. HRMEC were stimulated at 37°C for 5 to 90 min. Subsequently, cells were washed 3 times with ice-cold PBS to stop the induction and lysis buffer was added. Cells were lysed in 6 M ureum, 1 mM ethylenediaminetetraacetic acid (EDTA), 0.5% Triton X-100, 5 mM NaF in PBS (pH 7,2–7,4) complemented with protease and phosphatase inhibitors. Lysates were cleared by centrifugation (10 min, 400 g, 4°C) and divided into three aliquots per lysate. Each aliquot was tested only once, immediately after thawing on ice. Concentrations of the phosphorylated and activated form of ERK1/2 were determined using ELISA [DuoSet® IC ELISA for phospho-ERK1 (Thr202/Tyr204) plus phospho-ERK2 (Thr185/Tyr187) from R&D Systems]. Simultaneously, total protein content was determined in a bicinchoninic acid (BCA) protein assay (Pierce, Rockford, IL).

### Matrigel Assay

Network formation in response to NT-3 and NT-4 was investigated using BD Matrigel basement membrane matrix with reduced growth factor content (BD Biosciences, Bedford, MA, USA). IBIDI µ-slides for angiogenesis were coated with Matrigel (IBIDI, Planegg, Germany) which was allowed to solidify for 30 min at 37°C. Subsequently, HRMEC in 50 µL of EBM-2 plus 0.5% of BSA were seeded (10000 cells/well) and incubated with NT-3 or NT-4 at 37°C. Each peptide was tested at different concentrations in triplicate. In at least three control wells per test plate dilution medium was added. Tube formation was monitored every hour with transmitted light by using an Axiovert 200 M inverted microscope, equipped with an EC Plan-Neofluar 10×/0.30 dry objective and a XL-3 incubator. Pictures were taken with an AxioCam MRm camera and processed with AxioVision software release 4.6.3 (Zeiss). For each experiment, the time point chosen for evaluation was the minimal incubation period necessary for optimal tube formation under our experimental conditions (11–15 h after seeding).

### Statistical Analysis

The non-parametric Mann-Whitney test was used to compare means from two independent groups. Pearson correlation coefficients were computed to investigate correlations between variables. A p-value less than 0.05 indicated statistical significance. SPSS version 12.0 and program 3S from the BMDP 2007 Statistical Package were used for the statistical analyses.

## Results

### Levels of Neurotrophins and Neurotrophin Receptors in Vitreous Samples

With the use of the Western blot analysis we demonstrated that NT-3, NT-4, TrkA, and TrkB were detected in all vitreous samples from patients with PDR and at lower levels in control patients without diabetes. On the other hand, NGF, BDNF and TrkC were not detected in vitreous samples from patients with PDR and nondiabetic control patients. TrkA and TrkB proteins migrated as several protein bands upon SDS-PAGE when immunoblotted and analyzed with the specific mouse monoclonal antibodies (Fig. 1). The intact receptor originated most probably from debris after cell death, whereas the major amounts of receptor immunoreactivity originated from proteolytic fragments, also dubbed soluble receptor fragments. In our analysis, the upper band of TrkA corresponded to the intact protein and was used for densitometric analysis, whereas the much more abundant lower protein bands corresponded to cleaved TrkA truncation forms (Fig. 1, Panel A). Intact TrkB, as evaluated by molecular weight standardization, was more abundant in vitreous of diabetic patients than in control vitreous. Again, various truncation forms were observed, mainly in diabetic vitreous samples (Fig. 1, Panel B). Densitometric analysis of the bands demonstrated a significant increase in NT-3 (p<0.001, Mann-Whitney test), NT-4 (p<0.001, Mann-Whitney test), TrkA (p = 0.049, Mann-Whitney test), and TrkB (p = 0.003, Mann-Whitney test) expression in vitreous samples from PDR patients compared to control patients (Fig. 2). Upon standardization for protein content, the expression levels of NT-3 and Trk-A were significantly higher in vitreous samples compared with paired serum samples from patients with PDR (p<0.001 for both comparisons, Mann-Whitney test) (Fig. 3). With the use of ELISA, we confirmed that NGF, and BDNF were not detected in vitreous samples from patients with PDR and nondiabetic control patients.

**Figure 1:** Examples of Western blot analysis of TrkA and TrkB in random human vitreous samples from 3 patients with proliferative diabetic retinopathy (D) and 3 control patients without diabetes (C). A representative set of samples is shown. Equivalent amounts of vitreous samples were separated by SDS-PAGE in a 12% acrylamide gel, blotted to a nitrocellulose membrane and then probed with a monoclonal antibody against TrkA (panel A) and TrkB (panel B). At the right side a molecular weight marker was included and the migration of known proteins is indicated in kilodaltons (kDa). The arrow indicates the intact protein and the lower bands correspond to cleaved TrkA and TrkB fragments.

**Figure 2:** Comparisons of mean band intensities for neurotrophin-3 (NT-3), neurotrophin-4 (NT-4), TrkA, and TrkB in vitreous samples from proliferative diabetic retinopathy (PDR) patients (n = 16) and nondiabetic control patients (n = 15). *The difference between the two means was statistically significant at 5% level.

**Figure 3:** Comparisons of mean band intensities for neurotrophin-3 (NT-3) (A) and TrkA (B) in equal amounts of protein from paired vitreous and serum samples from patients with proliferative diabetic retinopathy (n = 12). *The difference between the two means was statistically significant at 5% level.

### Immunohistochemical Analysis

No staining was observed in the negative control slides (Fig. 4A). All membranes showed blood vessels positive for the panendothelial cell marker CD34 (Fig. 4B), with a mean number of 69.3±68.8 (range, 12–270). Immunoreactivity for NT-3 was present in all membranes and was noted in the cytoplasm of stromal cells and vascular endothelial cells (Fig. 4D, E). The number of immunoreactive stromal cells ranged from 18 to 190, with a mean number of 78.2±50.2. The number of immunoreactive blood vessels ranged from 2 to 46, with a mean number of 12.5±11.5. No immunoreactivity was observed for NT-4. Cytoplasmic immunoreactivity for TrkA, TrkB, and TrkC was present in stromal cells and vascular endothelial cells in all membranes (Fig. 5). The number of stromal cells immunoreactive for TrkA ranged from 15 to 175, with a mean number of 71.9±43.1. The number of blood vessels immunoreactive for TrkA ranged from 4 to 30, with a mean number of 16.6±8.5. The number of stromal cells immunoreactive for TrkB ranged from 33 to 200, with a mean number of 92.4±55.1. The number of blood vessels immunoreactive for TrkB ranged from 2 to 25, with a mean number of 12.7±7.4. The number of stromal cells immunoreactive for TrkC ranged from 20 to 180, with a mean number 62.2±45.1 The number of blood vessels immunoreactive for TrkC ranged from 0 to 28, with a mean number of 12.7±9.2. In serial sections, the distribution of myofibroblasts expressing α-SMA (Fig. 4C) was similar to the distribution of stromal cells expressing NT-3, TrkA, TrkB, and TrkC.

**Figure 4:** Proliferative diabetic retinopathy epiretinal membranes. Negative control slide that was treated with an irrelevant antibody showing no labeling (A) (original magnification×40). Immunohistochemical staining for CD34 showing blood vessels positive for CD34 (B) (original magnification×40). Immunohistochemical staining for α-smooth muscle actin showing immunoreactivity in spindle-shaped myofibroblasts (C) (original magnification×100). Immunohistochemical staining for neurotrophin-3 showing vascular endothelial cells (arrows) (D) and stromal cells (arrowheads) (E) expressing immunoreactivity for neurotrophin-3 (original magnification×100).

**Figure 5:** Proliferative diabetic retinopathy epiretinal membranes. Immunohistochemical staining for TrkA. Low power (A) (original magnification×40) and high power (B, C) (original magnification×100) showing vascular endothelial cells (arrows) and stromal cells (arrowheads) expressing TrkA. Immunohistochemical staining for TrkB. Low power (D) (original magnification×40) and high power (E) (original magnification×100) showing immunoreactivity in vascular endothelial cells (arrows) and stromal cells (arrowheads). Immunohistochemical staining for TrkC. Low power (F) (original magnification×40) and high power (G, H) (original magnification×100) showing vascular endothelial cells (arrows) and stromal cells (arrowheads) expressing TrkC.

### Correlations and Relationship with PDR Activity

The mean numbers of blood vessels expressing CD34, were significantly higher in membranes from patients with active PDR than in membranes from patients with inactive PDR. In addition, the mean numbers of stromal cells expressing NT-3, TrkA, TrkB, and TrkC were significantly higher in membranes from patients with active PDR than in membranes from patients with inactive PDR (Table 2).

**Table 2:** Mean numbers of immunoreactive blood vessels and stromal cells in epiretinal membranes in relation to type of proliferative diabetic retinopathy (PDR).

Variable	Active PDR(n = 8)Mean ± SD	Inactive PDR(n = 10)Mean ± SD	p-value(Mann-Whitney test)
• Blood vessels expressing CD34	110.3±83.5	32.9±14.0	0.001*
• Blood vessels expressing neurotrophin-3	13.5±9.6	11.7±13.5	0.529
• Cells expressing neurotrophin-3	111.9±48.6	48.3±29.0	0.003*
• Blood vessels expressing TrkA	19.8±10.0	13.4±5.8	0.092
• Cells expressing TrkA	96.9±44.6	46.9±23.8	0.015*
• Blood vessels expressing TrkB	13.9±8.3	11.6±6.8	0.469
• Cells expressing TrkB	126.9±52.0	61.7±38.1	0.014*
• Blood vessels expressing TrkC	16.9±8.1	8.5±8.6	0.073
• Cells expressing TrkC	85.8±50.9	38.6±22.6	0.011*

* Statistically significant at 5% level of significance.

The level of vascularization and proliferative activity in epiretinal membranes were determined by immunodetection of the panendothelial cells marker CD34. Significant correlations were detected between the number of blood vessels expressing CD34 and the number of blood vessels expressing TrkA (r = 0.571, p = 0.021). Furthermore, significant correlations were observed between the number of blood vessels expressing CD34 and the numbers of stromal cells expressing NT-3 (r = 0.559, p = 0.02), TrkA (r = 0.686, p = 0.003), TrkB (r = 0.643, p = 0.005), and TrkC (r = 0.722, p = 0.002).

### Effect of Diabetes on Retinal Expression of Neurotrophins and Neurotrophin Receptors in Experimental Rats

The previous clinical findings were corroborated in a preclinical diabetes rat model. We quantified the expression of NT-3, NT-4, TrkA, TrkB and TrkC in rat retinas by Western blot analysis. Densitometric analysis of the bands revealed a significant increase in NT-3, NT-4, TrkA, and TrkB (p<0.025 for all comparisons, Mann-Whitney test) in diabetic retinas compared to nondiabetic controls. On the other hand, the expression levels of TrkC did not differ significantly between diabetic and nondiabetic controls (Fig. 6).

**Figure 6:** Comparison of mean band intensity ratios for neurotrophin-3 (NT-3), neurotrophin-4 (NT-4), TrkA, TrkB and TrkC in the retinas of diabetic and control rats. Each Western blot experiment was repeated 3 times with fresh samples. *The difference between the two means was statistically significant at 5% level.

### Interactions of NT-3 and TrkA and TrkB

Co-immunoprecipitation studies were performed on 12-week-old diabetic rat retinas. Retinas were homogenized and homogenates were immunoprecipitated with an antibody against NT-3. The resulting immune complexes were analyzed by Western blot with antibodies against TrkA and TrkB. In the retinas of diabetic rats, NT-3 positively interacted with the receptors TrkA and TrkB (Fig. 7).

**Figure 7:** Co-immunoprecipitation assay to demonstrate interactions between neurotrophin-3 (NT-3) and the neurotrophin receptors TrkA and TrkB in the retinas of diabetic rats. The NT-3 band was immunoprecipitated within a complex between ligand and receptors. The TrkA and TrkB bands, present in the immunoprecipitates with an NT-33-reactive antibody, represent the interaction between NT-3 and the receptors TrkA and TrkB in diabetic (D) and control (C) rats.

### In vitro Angiogenic Activity of NT-3 and NT-4

Several studies report that neurotrophins have the potential to induce new vessel outgrowth. In view of their observed expression in PDR, we investigated whether NT-3 and NT-4 activate retinal microvascular endothelial cells in two experimental set-ups routinely used in our laboratory for this purpose, i.e. induction of ERK phosphorylation and network formation in matrigel. First, we performed four independent signaling assays and generated dose response curves for NT-3 and NT-4 (10–100 ng/ml) at 5 and 15 min after cell stimulation. Figure 8A shows that 15 min after stimulation no statistical significant induction of ERK phosphorylation was detected. Similarly, stimulation of HRMEC during 5 min did not increase ERK activation (data not shown). In contrast, VEGF at 10 ng/ml significantly raised the levels of phosphorylated ERK1/2 in HRMEC. In addition, we prolonged the stimulation period for treatment with 100 ng/ml of NT-3 and NT-4 to 90 min, but could not detect significant activation of ERK1/2 at any time point (Figure 8B). Next, we analyzed possible stimulatory activity of NT-3 and NT-4 on endothelial cells seeded on matrigel (n = 2). Endothelial cell migration in the presence of NT-3 and NT-4 (10–300 ng/ml) was monitored during 17 h. No clear angiogenic activity for NT-3 or NT-4 nor for 10 ng/ml of NGF (used as an additional internal control) was observed (data not shown).

**Figure 8:** Human retinal microvascular endothelial cells were stimulated with neurotrophin-3 (NT-3), neurotrophin-4 (NT-4) or vascular endothelial growth factor (VEGF) to induce phosphorylation of extracellular signal regulated kinase (ERK). Results were expressed relative to the phosphorylation level of ERK after stimulation with dilution medium (Control). (A) In the upper panel, data are shown from cells that were stimulated for 15 minutes with 10 to 100 ng/ml of NT-3 or NT-4 or 10 ng/ml of VEGF. (B) In the lower panel, we visualize the effects of a fixed concentration of NT-3 or NT-4 (100 ng/ml) added to the endothelial cells. The cells were lysed after 5, 15, 45 or 90 minutes and ERK phosphorylation as evaluated. Values are averages from 1 to 4 experiments ± SEM. * indicates significantly enhanced ERK phosphorylation (Mann-Whitney test).

## Discussion

The present study provides evidence for increased local levels of NT-3 and NT-4 in the vitreous fluid from patients with PDR as compared to nondiabetic control patients, whereas NGF and BDNF were undetectable in both diabetic patients and controls. This study also described for the first time, the *in situ* localization of the expression of NT-3 and the neutrophin receptors TrkA, TrkB, and TrkC in epiretinal membranes from patients with PDR. On the other hand NT-4 was not detected. Furthermore, we demonstrated upregulated expression of NT-3 and NT-4 and their receptors TrkA and TrkB, but not of TrkC in the retinas of diabetic rats. The levels of the NTs and their receptors in vitreous samples were significantly higher than the serum levels. Moreover, NTs and their receptors were expressed in PDR fibrovascular epiretinal membranes. These findings suggest that local cellular production is the relevant source of these ligands within the ocular microenvironment and that NT-3 and NT-4 and their receptors may be associated with the progression of PDR.

In the present study, we showed that NT-3 and NT-4 expression was upregulated in the vitreous fluid from patients with PDR, whereas NGF and BDNF levels were below the detection limit of our test system. In addition, we demonstrated upregulation of NT-3 and NT-4 in the retinas of diabetic rats. In contrast to a previous study in which elevated levels of NGF were detected in the vitreous fluid from patients with idiopathic epiretinal membranes [21], NGF was not detected in the vitreous in our study. Reasons for this discrepancy are not obvious, but two different methods were used to assess the expression of NGF in our study. Our results of increased levels of NT-3 and NT-4 in the vitreous samples from patients with PDR and upregulation of NT-3 and NT-4 in the retinas of diabetic rats are consistent with previous reports showing that NT-3 and NT-4 play a role in the development of diabetic complications. NT-3 mRNA was upregulated in the dorsal root and sural nerve of 12-week streptozotocin-diabetic rats [22]. NT-3 protein is also increased in the skin from patients with diabetic neuropathy [23]. In addition, the expression of NT-3 and NT-4 is increased in the cavernous tissue in penises of streptozotocin-induced diabetic rats [24]. Other studies reported increased tear NGF levels in patients with PDR [25] and that NGF treatment of diabetic rats prevented both neuroretinal programmed cell death and capillary pathology [26]. It was also demonstrated that diabetes-induced peroxynitrite mediates retinal neurodegeneration by inhibiting NGF survival signaling [27].

NTs and their corresponding receptors are not only expressed within the nervous system, but are also present in non-neuronal cells [5]–[11]. Another aim of the present study was to determine which cell types express NTs and their tyrosine kinase receptors TrkA, TrkB, and TrkC in epiretinal membranes from patients with PDR. Using immuno-histochemistry, we demonstrated for the first time that NT-3, TrkA, TrkB, and TrkC proteins were specifically localized in vascular endothelial cells and α-SMA-expressing myofibroblasts, whereas NT-4 was not detected. In addition, we found significant correlations between the level of vascularization in PDR epiretinal membranes and the number of blood vessels expressing TrkA and stromal cells expressing NT-3, TrkA, TrkB, and TrkC. The numbers of stromal cells expressing NT-3, TrkA, TrkB, and TrkC in membranes from patients with active PDR were significantly higher than those in membranes from patients with inactive PDR. The expression of TrkA, TrkB, and TrkC by endothelial cells in PDR epiretinal membranes suggests that these cells might be responsive to NT-3 and NT-4. In addition, increased levels of NT-3 and NT-4 in the vitreous fluid from patients with PDR and co-expression of NT-3 and its tyrosine kinase receptors in PDR epiretinal membranes suggest that they are associated with the progression of PDR. Despite the lack of expression of NT-4 in PDR epiretinal membranes, we could detect increased expression of NT-4 in the vitreous fluid from PDR patients and in the retinas of diabetic rats. This indicates that NT-4 might be of relevance in PDR progression. Our *in vivo* data are in agreement with previous *in vitro* studies that demonstrated expression of neurotrophin receptors by several endothelial cell types [5], [28]–[30] and that myofibroblasts synthesize and secrete NT-3 and express TrkA, TrkB, and TrkC [6]. These findings suggest that myofibroblasts participate in the neurotrophin network not only by releasing neurotrophins but also by responding to their action. *In vivo* studies demonstrated immunoreactivity for NT-3 and Trk receptors in vessel walls, and stromal fibroblasts of lung cancer specimens [11]. In addition, TrkA expression and activation are increased in the kidneys from patients with diabetic nephropathy [31], and TrkA and TrkC expression is increased in human diabetic skin [32]. Our Western blot analysis demonstrated the presence of intact and cleaved TrkA and TrkB in the vitreous from PDR patients. Our findings are consistent with a previous study that demonstrated proteolytic cleavage of the cell membrane-bound TrkA receptor by the action of membrane-bound metalloprotease activities through a process called ectodomain shedding, releasing soluble extracellular domains. These findings explain the recovery of the ectodomain of TrkA and TrkB in the vitreous and as a soluble fragment from the culture media of cells [33]. Furthermore, we interpret the presence of intact Trks in the vitreous as originating from dead cells.

Recent studies provide evidence for a direct involvement of NTs in the angiogenic process, in addition to the well established role of angiogenic growth factors, such as VEGF [5], [12]–[17]. In a recent study, the proangiogenic potential of NT-3 was demonstrated. NT-3 stimulated human umbilical vein endothelial cell proliferation, survival, migration, and network formation on the basement membrane matrix Matrigel. *In vivo* studies demonstrated that levels of both NT-3 and phosphorylated TrkC increased in response to ischemia and that NT-3 is able to promote angiogenesis and to enhance reparative angiogenesis and, thus, enhance blood supply to ischemic limbs [5]. It was also reported that NT-3 secreted by gliomas is able to stimulate the migration of marrow stromal cells suggesting that NT-3 plays a role in tumor angiogenesis [17]. In addition, NT-4 was shown to promote neovascularization in an *in vivo* Matrigel implant model. NT-4-induced angiogenesis was as potent as that induced by VEGF [12]. Furthermore, TrkA overexpression enhanced tumor growth, angiogenesis, and metastasis of breast cancer cells [34]. However, when we evaluated the response of primary retinal endothelial cells to NT-3 and NT-4 *in vitro*, we could not confirm the angiogenic activity of these NTs. In the present study, VEGF induced significant ERK1/2 phosphorylation in retinal microvascular endothelial cells. On the other hand, NT-3 and NT-4 did not elicit phosphorylation of ERK1/2 and did not induce network formation in Matrigel. Our *in vitro* findings do not exclude the possibility that the NTs may have effects on other cell types or on endothelial cells from a different origin.

Several studies reported that NTs modulate fibroblast functions and could be involved in tissue remodeling, wound healing and fibrosis [6]–[9], [18]. Fibroblasts and myofibroblasts express the neurotrophin receptors TrkA, TrkB, and TrkC and NTs, including NT-3 and NT-4, promote fibroblast survival, migration and differentiation of fibroblasts into α-SMA-expressing myofibroblasts [6]. Moreover, increased expression of NT-4 and its cognate receptor TrkB was observed in human lungs explanted from patients with idiopathic pulmonary fibrosis, and in lungs from mice with bleomycin-induced pulmonary fibrosis [10].

In conclusion, the data reported in the present study suggest that the NT-3 and NT-4/Trk axis is upregulated in the ocular microenvironment in patients with PDR and is associated with the progression of PDR. Further studies are required to explore the functional role played by this pathway in the pathogenesis of angiogenesis and fibrosis associated with PDR.
